The article "Intelligent Algorithm-Based Ultrasound Image for Evaluating the Effect of Comprehensive Nursing Scheme on Patients with Diabetic Kidney Disease" was published in 2022. Journal: Comput Math Methods Med.

# Intelligent Algorithm-Based Ultrasound Image for Evaluating the Effect of Comprehensive Nursing Scheme on Patients with Diabetic Kidney Disease

**DOI:** 10.1155/2022/6440138

**Published:** 2022-03-10

**Authors:** Chunyan Zhao, Qiuyu Shi, Fuying Ma, Junjuan Yu, Aijuan Zhao

**Affiliations:** ^1^Department of Renal Medicine, The First Affiliated Hospital of Jiamusi University, Jiamusi, 154002 Heilongjiang, China; ^2^Department of Endocrinology, The First Affiliated Hospital of Jiamusi University, Jiamusi, 154002 Heilongjiang, China; ^3^Ministry of Medical and Continuing Education after Graduation, The First Affiliated Hospital of Jiamusi University, Jiamusi, 154002 Heilongjiang, China

## Abstract

This study was aimed at exploring the effect of ultrasound image evaluation of comprehensive nursing scheme based on artificial intelligence algorithms on patients with diabetic kidney disease (DKD). 44 patients diagnosed with DKD were randomly divided into two groups: group A (no nursing intervention) and group B (comprehensive nursing). In the same period, 32 healthy volunteers were selected as the control group. Ultrasonographic images based on the *K* non-local-means (KNL-Means) filtering algorithm were used to perform imaging examinations in healthy people and DKD patients before and after care. The results suggested that compared with those of the SAE reconstruction algorithm and KAVD reconstruction algorithm, the PSNR value of artificial bee colony algorithm reconstruction of image was higher and the MSE value was lower. The resistant index (RI) of DKD patients in group B after nursing was 0.63 ± 0.06, apparently distinct from the RI of the healthy people (controls) in the same group (0.58 ± 0.06) and the RI of DKD patients in group A (0.68 ± 0.07) (*P* < 0.05). The incidence rate of complications in DKD patients in group B was apparently inferior to that in group A. After comprehensive nursing intervention (CNI), the scores of all dimensions of quality of life (QoL) in DKD patients in group B were obviously superior versus those in DKD patients in group A. It suggests that implementation of nursing intervention for DKD patients can effectively help patients improve and control the level of renal function, while ultrasound images based on intelligent algorithm can dynamically detect the changes in the level of renal function in patients, which has the value of clinical promotion.

## 1. Introduction

Diabetes mellitus (DM), a common disease with high incidence in clinical practice [1], has rapidly increased its prevalence with improved people's living standards in recent years. At present, China is the country with the highest total number of DM worldwide. Diabetic kidney disease (DKD), a chronic kidney disease (CKD) caused by long-term progression of DM, is one of the most likely and serious microvascular diseases among the complications of DM and one of the main factors leading to end-stage renal disease (ESRD) [2]. DKD is a systemic disease with chronic hyperglycemia as the main clinical feature, which causes glucose, protein, and fat metabolism disorders due to absolute or relative insulin deficiency in the body under different pathogenic factors and pathogenesis [3]. DM damages various tissues in the kidney through different pathways, of which only glomerulosclerosis and DM are directly related, so it is known as DKD and is a kind of systemic microvascular complication of DM [4]. Clinical manifestations include hypertension, advanced severe renal failure, progressive renal damage, edema, and proteinuria, which is one of the main causes of death in DKD patients [5].

The article "Intelligent Algorithm-Based Ultrasound Image for Evaluating the Effect of Comprehensive Nursing Scheme on Patients with Diabetic Kidney Disease" was published in 2022. Journal: Comput Math Methods Med.

The treatment of DKD lacks effective methods, so once DM patients have complicated kidney damage, the condition tends to be progressive, until uremia [6]. Clinical nursing can control the process of disease, improving the survival ability of patients, which is an important part of the treatment of DKD [7]. DKD is a common complication of DM. With the progression of the disease, it is easy to develop into ESRD. Clinical studies found that effective nursing intervention for patients with DKD can be carried out through psychological nursing, infection prevention, health education, patient behavior nursing intervention, drug nursing, and diet nursing. It can improve patients' understanding of DKD knowledge, clarify the harm of DKD, face up to the treatment of disease positively, correct bad life and eating habits, establish a correct and healthy attitude to life, improve the coordination of clinical medication and treatment, respond to disease with positive and good psychological and physiological conditions, and help patients to promote recovery of the disease. It also helps to improve the quality of nursing [8].

With the emergence and continuous development of ultrasonic diagnosis technology, it is possible to dynamically monitor the generation, development, and prognosis of DKD [9]. Ultrasound is a convenient, fast, noninvasive, and efficient imaging method. It can not only directly display the shape and size of the kidney, vascular morphology, parenchymal echo, and other physiological data but also combine with color imaging and spectral Doppler. It can dynamically monitor the progressive branches of renal artery and blood perfusion in real time and provide hemodynamic parameter information [10]. In recent years, with the continuous development of ultrasonic technology and ultrasonic equipment, more and more new technologies are gradually popularized and used in clinical practice. However, speckle noise is often present in ultrasonography images [11], which can cause loss of structural information in the image. At present, the study of denoising methods for ultrasonic images has become the focus of attention. Some studies put forward that the nonlocal means (NL-Means) filtering algorithm has good effect for denoising, but it cannot well preserve the details of the image and the edge information [12]. Therefore, some experts presented the idea of clustering—*K*-means clustering (K-Means) [13], which classifies and sorts the images that need to be processed and then uses the NL-Means filtering algorithm for denoising processing. The research results indicate that the NL-Means algorithm based on *K*-means clustering (abbreviated as KNL-Means) solves the problem of image details and edge information retention and has a good application effect [14].

The article "Intelligent Algorithm-Based Ultrasound Image for Evaluating the Effect of Comprehensive Nursing Scheme on Patients with Diabetic Kidney Disease" was published in 2022. Journal: Comput Math Methods Med.

Therefore, the artificial bee colony algorithm was used to screen the eigenvalues of kidney images, reduce the feature latitude, shorten the time of classification and training, and weaken the complexity of calculation. In addition, the artificial bee colony algorithm was used to find the optimal parameters needed to support the classification of ultrasound images, so as to improve the accuracy of classification. The patients with DKD after nursing intervention were examined to explore the effect of nursing intervention on DKD patients, providing data support for subsequent clinical applications.

## 2. Research Methods

### 2.1. Study Subjects

In this study, data from 44 patients with DKD admitted to hospital from June 2019 to April 2020 were collected, including 28 males (average age of 55.74 ± 12.82), aged 28~83 years, and 16 females, aged 35~79 years (56.91 ± 10.27), with 24 patients with a disease course of 1-5 years and 20 patients of 6-20 years. The patients were randomly divided into two groups: group A (no nursing intervention) and group B (comprehensive nursing). In the same period, 32 healthy volunteers of similar age were selected as the healthy controls (control group), including 18 males and 14 females, aged 23~66 years (41.38 ± 10.73). Imaging examination was performed in healthy people and two groups of patients with DKD using ultrasound based on the intelligent algorithm. This study had been approved by the ethics committee of hospital, and the family members of the patients signed the informed consent form.

The following are the inclusion criteria: (1) patients who meet the diagnostic criteria of DKD and (2) informed consent of patients and patients' participation are voluntary. The following are the exclusion criteria: (1) combination of ketoacidosis and other acute complications of DM and (2) renal developmental defects, nephrotic syndrome, urinary system inflammation, acute nephritis, chronic nephritis, renal artery stenosis, hypertension, hyperlipidemia, obstruction and occupying lesions, and other diseases that may cause renal impairment; (3) hyperglycemia, hypertension, infection, fever, and strenuous exercise within 24 hours that may affect the accuracy of urinary albumin/creatinine ratio results; and (4) other serious systemic diseases.

The article "Intelligent Algorithm-Based Ultrasound Image for Evaluating the Effect of Comprehensive Nursing Scheme on Patients with Diabetic Kidney Disease" was published in 2022. Journal: Comput Math Methods Med.

### 2.2. Nursing Interventions

The following are the nursing interventions:

- Psychological nursing: long-term illness and treatment bring great economic pressure and psychological burden to patients, which easily lead to anxiety, hopelessness, helplessness, and other negative emotions. Nursing staff need to care for patients in time, help patients establish confidence to overcome the disease, correctly understand and treat the disease, actively prevent and cooperate with the treatment, maintain continuous optimism, and reduce the negative emotions of patients.
- Medication nursing: the nursing staff should be familiar with the indications and contraindications of commonly used drugs in the treatment of DKD. During medication, the vital signs, skin color, mental status, urine protein, urine volume, and blood glucose of the patients should be closely observed and recorded.
- Skin care: the sugar content in the skin of patients with DKD is much higher versus that of normal people, and its environment is suitable for bacterial growth and breeding. When the blood glucose is high, the effect of phagocytes on bacterial phagocytosis is decreased, and the resistance to infection is reduced, so it often leads to patients with skin suppurative infection or fungal infection. The nursing staff should strengthen the nursing care of the patient's skin, maintain the skin in a dry and clean state, and instruct the patient to bathe frequently and change clothes frequently. For the patients who stay in bed for a long time, they should be scrubbed every other day, and the nursing staff need to pay attention to gentle movements. Moreover, due to DKD patients with long-term hypoproteinemia, they are easy to produce edema, and edema and neuropathy caused by small vessel disease are prone to cause skin damage.
- Diet nursing: healthy diet has an important impact on patients with DKD, so nursing staff should pay attention to the diet treatment of patients with DKD. The principle of treatment is to control dietary calories and adjust the proportion of nutrients appropriately. Besides reducing the burden of insulin B cells, it is also necessary to ensure the normal metabolic operation of the body.
- Others: patients with DKD should rest in bed until clinical symptoms disappear and urinalysis is normal. Patients in the recovery period can move appropriately but pay attention not to overexertion, arrange routines reasonably, and pay attention to keep warm, not causing aggravation or recurrence of the disease. Because obesity easily leads to lipid deposition on the glomeruli, which leads to deterioration of renal function, obese individuals should appropriately increase exercise to lose weight.
- Evaluation indicators: the incidence of complications in the two groups was compared and analyzed, and the SF-36 quality of life (QoL) scale was adopted to evaluate the QoL of the two groups. The higher the score, the better the QoL.

The article "Intelligent Algorithm-Based Ultrasound Image for Evaluating the Effect of Comprehensive Nursing Scheme on Patients with Diabetic Kidney Disease" was published in 2022. Journal: Comput Math Methods Med.

### 2.3. Ultrasonic Evaluation

All subjects were examined by ultrasound on an empty stomach, in a supine position. Using color Doppler ultrasound diagnostic instrument for color Doppler measurement, C5-2 ultra-wideband probe was used. When the color blood flow signal of the renal artery was clearly displayed, the patient was required to hold his/her breath. The blood flow parameters of the renal aorta, the intrarenal artery, and the interlobar artery at the renal hilum were measured, that is, peak systolic blood flow velocity (PSV) and end diastolic blood flow velocity (EDV), and blood flow resistant index (RI) of the intrarenal artery was calculated. The calculation equation is RI = (PSV − DEV)/PSV.

### 2.4. NL-Means Denoising Algorithm

The NL-means denoising algorithm can reasonably utilize the redundant information in ultrasonic images to achieve good denoising effect [15]. It also makes weights more accurate by comparing pixels among all regions of the image. It is assumed that the ultrasound image containing speckle noise is *N*; *x*, *y*, *z* are pixels in the image, where the two-dimensional bounded region is set as *β* ∈ *R*^2^, *x*, *y*, *z* ∈ *β*; the algorithm is shown as

(1) $$\begin{array}{c} S\left(N\right)\left(x\right)=\frac{1}{M\left(x\right)}\times_{\beta }\int \exp\left[-\frac{G_{N}*{\left|N\left(x+.\right)-N\left(y+.\right)\right|}^{2}\left(0\right)}{h^{2}}\right]\times N\left(y\right)dy, \end{array}$$

(2) $$\begin{array}{c} \text{Means}\left(x\right){=}_{\beta }\int \exp\left[-\frac{G_{N}*{\left|N\left(x+.\right)-N\left(z+.\right)\right|}^{2}\left(0\right)}{h^{2}}\right]\times dz, \end{array}$$

(3) $$\begin{array}{c} G_{N}*{\left|N\left(x+.\right)-N\left(y+.\right)\right|}^{2}\left(0\right){=}_{R^{2}}\int G_{N}\left(l\right){\left|N\left(x+l\right)-N\left(y+l\right)\right|}^{2}dl. \end{array}$$

*S* represents any pixel in an ultrasound image, *G*_*n*_ means a Gaussian convolution kernel of *n*, *h* presents a filter coefficient, and *h* is obtained through the noise standard deviation of the ultrasound image itself.

The article "Intelligent Algorithm-Based Ultrasound Image for Evaluating the Effect of Comprehensive Nursing Scheme on Patients with Diabetic Kidney Disease" was published in 2022. Journal: Comput Math Methods Med.

For the discrete region, it is assumed that the discrete image is *w*, and *w* = {*w*(*i*), *i* ∈ *α*}. *α* represents the pixel set. Then, the NL-Means denoising algorithm is expressed as

(4) $$\begin{array}{c} S\left(w\right)\left(i\right)=\underset{j\in \alpha }{\sum }T\left(i,j\right)w\left(j\right), \end{array}$$

(5) $$\begin{array}{c} T\left(i,j\right)=\frac{1}{K\left(i\right)}\exp\left[-\frac{{\left\|w\left(W_{i}\right)-w\left(W_{j}\right)\right\|}_{2a}^{2}}{h^{2}}\right], \end{array}$$

(6) $$\begin{array}{c} K\left(i\right)=\underset{j}{\sum }\exp\left[-\frac{{\left\|w\left(W_{i}\right)-w\left(W_{j}\right)\right\|}_{2a}^{2}}{h^{2}}\right]. \end{array}$$

*T* means the distance of image neighborhood, and *K* is the discrete coefficient of image. However, the above method will introduce artificial artifacts in the process of image processing, so it is necessary to add image gradient information to effectively solve this problem. When image gradient information is supplemented to NL-means, the expression changes.

Algorithm representation of ultrasonic image *N* with speckle noise is shown as

(7) $$\begin{array}{c} S\left(N\right)\left(x\right)=\frac{1}{M\left(x\right)}\times_{\beta }\int \exp\left\{-\frac{\left[G_{N}*{\left|N\left(x+.\right)-N\left(y+.\right)\times \left(\Delta N\left(x+.\right)-\Delta N\left(y+.\right)\right)\right|}^{2}\left(0\right)\right]}{h^{2}}\right\}\times n\left(y\right)dy, \end{array}$$

(8) $$\begin{array}{c} \text{Means}\left(x\right){=}_{\beta }\int \exp\left\{-\frac{\left[\left(G_{N}*{\left|N\left(\text{x}+.\right)-N\left(z+.\right)\times \Delta N\left(\text{x}+.\right)-\Delta N\left(z+.\right)\right|}^{2}\right)\left(0\right)\right]}{h^{2}}\right\}\times dz, \end{array}$$

(9) $$\begin{array}{c} \left(G_{N}*\right.{\left|\left.N\left(x+.\right)-N\left(y+.\right)\right)\times \left(\Delta N\left(x+.\right)-\Delta N\left(y+.\right)\right)\right|}^{2}\left(0\right){=}_{R^{2}}\int G_{N}\left(l\right){\left|\left(N\left(x+l\right)-N\left(y+l\right)\right)\times \left(\Delta N\left(x+l\right)-\Delta N\left(y+l\right)\right)\right|}^{2}dl. \end{array}$$

Algorithm representation of discrete image *w* is shown as

(10) $$\begin{array}{c} S\left(w\right)\left(i\right)=\underset{j\in \alpha }{\sum }T\left(i,j\right)w\left(j\right), \end{array}$$

(11) $$\begin{array}{c} T\left(i,j\right)=\frac{1}{K\left(i\right)}\exp\left[-\frac{{\left\|\left(w\left(W_{i}\right)-w\left(W_{j}\right)\right)\times \left(\Delta w\left(W_{i}\right)-\Delta w\left(W_{j}\right)\right)\right\|}_{2a}^{2}}{h^{2}}\right], \end{array}$$

(12) $$\begin{array}{c} K\left(i\right)=\underset{j}{\sum }\exp\left[-\frac{{\left\|\left(w\left(W_{i}\right)-w\left(W_{j}\right)\right)\times \left(\Delta w\left(W_{i}\right)-\Delta w\left(W_{j}\right)\right)\right\|}_{2a}^{2}}{h^{2}}\right]. \end{array}$$

Δ denotes image gradient information, which will reduce the correlation between adjacent images, so that the region with more image details has obviously reduced amplitude, while the region with relatively smooth image has slowly reduced amplitude. Then, increasing *h* and further smoothing, it is aimed at making artificial pseudo but also at preserving the detailed information of the image. However, because the denoising effect is not obvious, the *K*-means clustering algorithm is added.

The article "Intelligent Algorithm-Based Ultrasound Image for Evaluating the Effect of Comprehensive Nursing Scheme on Patients with Diabetic Kidney Disease" was published in 2022. Journal: Comput Math Methods Med.

### 2.5. NL-Means Denoising Algorithm Based on *K*-Means Clustering

*K*-means clustering is a method to indirectly aggregate and classify similar regions in images, which requires setting the cluster center and then classifying similar samples [16]. For the remaining objects, they were reasonably assigned by calculating their distance from the cluster center, after which the average was calculated as the cluster center. Clustering is stopped once the standard measure function begins to converge. This method is sensitive to isolated noise and will not affect the detailed information of the image itself. It is clearly helpful for the NL-Means denoising algorithm in denoising efficiency improvement [17, 18].

The K-means clustering algorithm steps are as follows.

(Step 1) *K* cluster centers are randomly selected in the target image, which are set as *u*_1_^(0)^, *u*_2_^(0)^, ⋯, *u*_*m*_^(0)^, *m* = 0, so the number of clusters in the image is *K*.
(Step 2) Objects {*x*_*i*_}(*i* = 1, 2, ⋯, C) in other regions are divided into the smallest distance class of *K*, that is, when $s_{il}^{\left(m\right)}=\underset{j}{\min}\left\{s_{il}^{\left(m\right)}\right\}\left(i=1,2,\cdots ,\text{C}\right)$ and *l* ∈ {1, 2, ⋯, *k*}, *x*_*i*_ ∈ *ω*_*l*_^(*m* + 1)^. *s*_*il*_^(*m*)^ presents the distance *u*_*j*_^(*m*)^ from *x*_*i*_ to *ω*_*j*_^(*m*)^, *m* means the number of iterations, and the generated clustering is expressed in

(13) $$\begin{array}{c} \omega_{j}^{\left(m+1\right)}\;\left(j=1,2,\cdots ,k\right). \end{array}$$

(Step 3) Various centers are calculated after reclassification, and the specific algorithm is shown in

(14) $$\begin{array}{c} u_{j}^{\left(m+1\right)}=\frac{1}{N_{j}^{\left(m+1\right)}}\underset{x_{i}\in \omega_{j}^{\left(m+1\right)}}{\sum }x_{i},\;j=1,2,..,k. \end{array}$$

*u*_*j*_^(*m* + 1)^ is the number of objects contained in the class *ω*_*j*_^(*m* + 1)^.

The article "Intelligent Algorithm-Based Ultrasound Image for Evaluating the Effect of Comprehensive Nursing Scheme on Patients with Diabetic Kidney Disease" was published in 2022. Journal: Comput Math Methods Med.

(Step 4) If *u*_*j*_^(*m* + 1)^ = *u*_*j*_^(*m*)^ (*j* = 1, 2, .., *k*), then the clustering ends, and if *u*_*j*_^(*m* + 1)^ ≠ *u*_*j*_^(*m*)^ (*j* = 1, 2, .., *k*), then *m* = *m* + 1, and the calculation is continued from Step 2.

### 2.6. Statistical Methods

SPSS22.0 data analysis software was applied. Measured values were represented as the mean ± standard deviation ($\overset{¯}{x}\pm s$), and count data was represented as percentage. Comparison between the two groups of measurement data was processed by a *t*-test, and a *t*-test and *x*^2^ test were adopted for analysis. When *P* < 0.05, the distinction had statistical significance.

## 3. Results

### 3.1. Algorithm Simulation Results

The test image is divided into 8 × 8 image blocks, and the denoising effect of the original image and K-means, NL-Means, and KNL-Means algorithm models is given in Figure 1. The corresponding comparison between PSNR and MSE is illustrated in Figures 2 and 3. The PSNR values of image reconstruction under SAE, K-SVD, and artificial bee colony algorithm models were 19.88 ± 4.11 dB, 24.95 ± 5.37 dB, and 29.37 ± 4.48 dB, respectively; MSE values were 0.0039 ± 0.0008, 0.0018 ± 0.0004, and 0.0016 ± 0.0005, respectively. By contrast, the image denoising effect of the KNL-Means algorithm model was distinctly better than that of K-means and NL-Means algorithms. The test revealed that the KNL-Means algorithm had good performance in ultrasonic image denoising processing.

### 3.2. Image Analysis of Renal Blood Flow in DKD Patients

The renal blood flow of DKD patients under algorithm-based ultrasound guidance is illustrated in Figure 4. Images can clearly reflect the kidney tissue structure (appearance like broad beans, local capsule uneven, not smooth, renal parenchymal thickness (>1 cm), normal echo, renal blood vessels, and renal pelvis can be complete and continuous display). Color Doppler showed that the renal blood flow filling state was slightly poor. Although the main renal artery and vein at the renal hilum could be displayed, its blood vessels were tortuous, and the renal blood flow signal gradually weakened. The diameters of the segmental artery and vein and the interlobar artery and vein entering the renal sinus were different, and the intrarenal artery suddenly narrowed and truncated. Doppler spectrum showed that the renal artery at the renal hilum was filled with blood flow during diastole, and the curve of spectrum during systole increased rapidly. The peak was blunt and incised and then decreased slowly, with frequency window filling.

The article "Intelligent Algorithm-Based Ultrasound Image for Evaluating the Effect of Comprehensive Nursing Scheme on Patients with Diabetic Kidney Disease" was published in 2022. Journal: Comput Math Methods Med.

### 3.3. Detection and Analysis of Renal Artery RI in DKD Patients

Figure 5 shows the changes of renal artery RI in healthy controls, group A, and group B. The RI value of DKD patients in group B after nursing was 0.63 ± 0.06, apparently distinct from those of the controls (0.58 ± 0.06) in the same group of healthy people (*P* < 0.05) and the DKD patients in group A (0.68 ± 0.07) (*P* < 0.05). According to the results, it can be inferred that the clinical nursing of patients with DKD helps to reduce the RI value, but there is still a difference in the RI value between patients with DKD and healthy people, indicating that comprehensive nursing can improve the renal artery high resistance of patients to a certain extent.

### 3.4. Contrast of Complications

According to the results of the study, the incidence of complications in patients with DKD in group B was only 27.28%, which was clearly inferior to that in group A. The distinction between the two groups had statistical significance (Figure 6).

### 3.5. QoL Score Comparison before and after Nursing

Before intervention, there was no significant difference in the scores of each dimension of QoL in two groups (*P* > 0.05). After comprehensive nursing intervention (CNI), the QoL scores of DKD patients in group B were distinctly better than those in group A (*P* < 0.05) (Figure 7).

## 4. Discussion

The main pathological mechanism of DKD is the obstruction of the glomerular interior and capillary network and the continuous thickening of the glomerular capillary basement membrane, resulting in hemodynamic changes and increased resistance to forward blood flow [19]. With the continuous development of the disease, it will eventually cause hemodynamic changes in renal arteries at all levels. Ultrasound based on an intelligent algorithm can repeatedly obtain the ultrasonic spectrum reflecting the changes of renal blood flow, which has helped to understand the changes of renal artery blood flow at all levels [20]. The results showed that compared with the SAE reconstruction algorithm and KAVD reconstruction algorithm, the PSNR value of the reconstructed image by the artificial bee colony algorithm was higher and the MSE value was lower. Through the comparison of PSNR and MSE of SAE reconstruction image, K-SVD reconstruction image, and artificial bee colony algorithm reconstruction image, it indicated that the image reconstruction effect of artificial bee colony algorithm model was significantly better than that of SAE reconstruction and KAVD reconstruction, and it had good performance in ultrasonic image reconstruction.

Renal ultrasound examination showed that the intrarenal blood flow signal was gradually weakened in DKD patients. Although the main renal artery could be clearly displayed, the diameter of intrarenal artery was different or narrowed, and there was sudden narrowing or truncation of intrarenal artery, which could indicate that with the continuous development of DM, the renal vascular damage was aggravated and the renal blood perfusion was gradually reduced. Moreover, the difference between RI of DKD patients in group A after nursing (0.63 ± 0.06) and that of the controls of the same group of healthy people (0.58 ± 0.06) had statistical meaning (*P* < 0.05), and the value (0.68 ± 0.07) before nursing was compared with that after nursing in group A; it had statistical difference. According to the results, it was inferred that RI decreased after clinical care for DKD patients, but there was still a difference in intrarenal RI values relative to healthy people, which indicated that comprehensive care could partially improve the renal artery high resistance status of patients. With the progression of renal impairment, gradual glomerular sclerosis, and renal vascular bed resistance gradually increasing, RI also further increased. RI and the course of DKD were positively correlated.

The article "Intelligent Algorithm-Based Ultrasound Image for Evaluating the Effect of Comprehensive Nursing Scheme on Patients with Diabetic Kidney Disease" was published in 2022. Journal: Comput Math Methods Med.

It was suggested that the scores of all dimensions of QoL in group B who had received CNI were apparently improved versus those in group A. Moreover, the incidence rate of complications in group B was 27.28%, apparently inferior than that in group A, indicating that CNI has a very significant effect on the improvement of the condition of patients with DKD, can reduce the probability of complications and promote improvement of the QoL and recovery of patients. In addition, because of the long course of DKD, in the treatment process, it is inevitable that depression, anxiety, and other negative emotions and even some patients will have the idea of suicide. For this reason, nursing staff need to try to understand the psychological changes of patients, conduct timely psychological intervention for patients, assist patients to get rid of negative emotions, improve the compliance of patients receiving treatment, and play an important role in the alleviation of doctor-patient disputes to a certain extent. In addition to psychological nursing intervention, the nursing staff should tell the patients to perform appropriate exercise, instruct the patients to perform appropriate exercise, enhance the patient's own physical fitness, and contribute to the improvement of the patient's condition. The nursing staff should also provide dietary guidance for the patients to ensure that the patients receive adequate nutrition, reduce the burden on the kidneys, and strengthen the nursing effect.

The article "Intelligent Algorithm-Based Ultrasound Image for Evaluating the Effect of Comprehensive Nursing Scheme on Patients with Diabetic Kidney Disease" was published in 2022. Journal: Comput Math Methods Med.

In conclusion, the use of CNI for patients with DKD has a very important role, which can reduce the complications of treatment, improve the QoL of patients, and contribute to the rehabilitation of patients and should be widely used in clinical practice. The increase of RI can be the evaluation standard of renal changes in DKD patients [21]. The ultrasound based on an intelligent algorithm can visually display the changes of intrarenal blood flow. Before the laboratory examination reveals obvious abnormalities, it can provide some reference value for the clinical diagnosis of DKD, so that most diabetic patients can obtain timely diagnosis and treatment at the reversible stage at the early stage of DKD disease and effectively control the development of the disease in time, thereby reducing the prevalence and mortality of DKD. It has a broad application and development prospect in clinic.

## 5. Conclusion

RI in diabetic patients is significantly higher than that in healthy people, which can be one of the diagnostic indicators of DKD. Nursing intervention can improve the high resistance state of renal artery to a certain extent. The addition of nursing intervention measures in the clinical treatment of DKD helps to improve the renal function level of patients, timely and effectively control, and promote the rehabilitation of patients. However, the sample size is small, and the accuracy of data needs further exploration. The denoising effect of ultrasonic image based on the KNL-Means algorithm is obviously superior, which can accurately detect the change of renal function level of patients. It can be used for auxiliary diagnostic measures and has further clinical popularization value.

## Figures and Tables

**Figure 1:** Reconstructed image results with different algorithms. (a) The original image of input; (b) the denoised image by the *K*-Means algorithm; (c) the denoised image by NL-Means algorithm; (d) the denoised image by the KNL-Means algorithm.

**Figure 2:** Comparison of simulation PSNR results of three reconstruction methods.

**Figure 3:** Comparison of simulation MSE results of three reconstruction methods.

**Figure 4:** Renal ultrasound blood flow of diabetic patients under comprehensive nursing.

**Figure 5:** Contrast of renal RI changes. ^∗^Compared to group A without comprehensive nursing, *P* < 0.05. ^#^Compared with healthy people, *P* < 0.05.

**Figure 6:** Incidence of complications in both groups. ^∗^Compared to group A, *P* < 0.05.

**Figure 7:** Contrast of QoL scores between the two groups. ^∗^Compared to group A, *P* < 0.05.

## Data Availability

The data used to support the findings of this study are available from the corresponding author upon request.
